The article "Ramentaceone, a Naphthoquinone Derived from Drosera sp., Induces Apoptosis by Suppressing PI3K/Akt Signaling in Breast Cancer Cells" was retracted in 2019. Reasons: duplicated images; original data or images not available; concerns about a third party's involvement.

# Ramentaceone, a Naphthoquinone Derived from *Drosera sp*., Induces Apoptosis by Suppressing PI3K/Akt Signaling in Breast Cancer Cells

**DOI:** 10.1371/journal.pone.0147718

**Published:** 2016-02-03

**Authors:** Anna Kawiak, Ewa Lojkowska

**Affiliations:** 1 Department of Biotechnology, Intercollegiate Faculty of Biotechnology, University of Gdansk and Medical University of Gdansk, Kladki 24, 80–822, Gdansk, Poland; 2 Laboratory of Human Physiology, Faculty of Health Sciences with Subfaculty of Nursing, Medical University of Gdansk, Tuwima 15, 80–210, Gdansk, Poland; University of Quebec at Trois-Rivieres, CANADA

## Abstract

The phosphoinositide 3-kinase (PI3K) signaling pathway plays an important role in processes critical for breast cancer progression and its upregulation confers increased resistance of cancer cells to chemotherapy and radiation. The present study aimed at determining the activity of ramentaceone, a constituent of species in the plant genera *Drosera*, toward breast cancer cells and defining the involvement of PI3K/Akt inhibition in ramentaceone-mediated cell death induction. The results showed that ramentaceone exhibited high antiproliferative activity toward breast cancer cells, in particular HER2-overexpressing breast cancer cells. The mode of cell death induced by ramentaceone was through apoptosis as determined by cytometric analysis of caspase activity and Annexin V staining. Apoptosis induction was found to be mediated by inhibition of PI3K/Akt signaling and through targeting its downstream anti-apoptotic effectors. Ramentaceone inhibited PI3-kinase activity, reduced the expression of the PI3K protein and inhibited the phosphorylation of the Akt protein in breast cancer cells. The expression of the anti-apoptotic Bcl-2 protein was decreased and the levels of the pro-apoptotic proteins, Bax and Bak, were elevated. Moreover, inhibition of PI3K and silencing of Akt expression increased the sensitivity of cells to ramentaceone-induced apoptosis. In conclusion, our results indicate that ramentaceone induces apoptosis in breast cancer cells through PI3K/Akt signaling inhibition. These findings suggest further investigation of ramentaceone as a potential therapeutic agent in breast cancer therapy, in particular HER2-positive breast cancer.

## Introduction

Breast cancer is one of the most frequently diagnosed malignancies in women and one of the leading causes of cancer-related deaths in the female population [1]. One of the major barriers in effective cancer treatment is the decreased potential of cancer cells to undergo apoptosis. One of the main regulators of apoptosis in breast cancer cells is the phosphoinositide 3-kinase (PI3K)/Akt pathway. PI3K/Akt signaling lies downstream of receptor tyrosine kinases and plays an important role among others in cellular metabolism, cell survival, proliferation and migration. Activation of the PI3K/Akt pathway has been associated with breast cancer development and confers resistance of breast cancer cells to conventional therapies, in particular HER2-directed therapy. HER2-overexpressing breast cancer accounts for 30% of breast cancer occurrences and is associated with increased resistance to chemotherapy, poor prognosis, and enhanced metastatic potential [2]. Several approaches aimed at targeting the HER2 receptor have been developed and include the application of monoclonal antibodies (e.g. trastuzumab) and tyrosine kinase inhibitors (e.g. lapatinib). Although therapies targeting the HER2 receptor have proven effective, patients do not respond equally to therapy and resistance is often acquired [3]. A combination of HER2 inhibition along with targeting a downstream molecule has been shown to increase the efficacy of HER2-overexpressing breast cancer treatment [4]. These findings warrant the search for new agents that target multiple components of the PI3K/Akt signaling pathway in order to achieve long-term inhibition of HER2-overexpressing tumors.

Ramentaceone (5-hydroxy-7-methyl-1,4-naphthoquinone) is a naphthoquinone present in plants of the Droseraceae family [5]. Ramentaceone has been found to display various biological activities such as antibacterial [6], [7], antifungal [8], and cytotoxic [9]. The cytotoxic activity of ramentaceone has been determined against different cell lines including murine lymphocytic leukemia (P-388) [10], human prostate cancer (LNCaP) [11] and human promyelocytic leukemia (HL-60) [12]. Our research regarding the effects of ramentaceone on leukemia HL-60 cells showed that ramentaceone induces cell death in HL-60 cells through the activation of the apoptotic machinery. Our recent research revealed that among the various cell lines examined, ramentaceone displayed high activity towards the breast cancer cell line, MCF-7 [9]. Due to the high activity of ramentaceone towards breast cancer cells, in our present study we focused on determining the mechanism of cell death induced by ramentaceone in breast cancer cells.

## Materials and Methods

### Extraction and isolation

The source of ramentaceone were 8-week-old plants obtained from *in vitro* grown cultures of *Drosera aliciae*. *D*. *aliciae in vitro* cultures were established from seeds obtained from the International carnivorous Plant Society Seed Bank (Pinole, CA, USA). Extraction and isolation of ramentaceone were performed according to the previously published procedures [12]. Briefly, dried plant material was sonicated at 50/60 Hz. Extracts were collected, evaporated and dissolved in chloroform. The obtained solution was evaporated on a rotovapour with coarse silica gel. Silica gel grains coated with the extract were loaded on silica gel column (150 g SiO_2_−60). Ramentaceone was isolated in a step gradient of methylene chloride in hexane from 50% to 100% of methylene chloride, concentration of methylene chloride was changed in 10% steps every 100 ml. 25 ml fractions were collected, combined and concentrated to dryness. The residue was dissolved in acetone and loaded to a LH-20 column. Fractions containing ramentaceone were combined and the procedure was repeated twice. Ramentaceone (PubChem CID: 26905) was obtained as yellow needles, mp 126°C, purity >97%, spectroscopic data: {NMR ^1^H (CDCl_3_): δ11.96 (1H, s, OH at C-5), δ 7.42 (1H, d, J = 2 Hz, H-2), δ 7.07 (1H, d, J = 2 Hz, H-3), δ 6.91 (2H, s, H-6 and H-8), δ 2.43 (3H, s, CH_3_ at C-7); high resolution ESI mass spectrometry: [M+H]^+^ at m/z 189.0555—registered and 189.055170—calculated for elemental composition: C_11_H_8_O_3_}. On the LC/UV chromatogram registered at λ = 280 nm a single peak was observed.

Melting points were determined with a Buchi melting point apparatus (model B-545). HPLC-ESI/MS analyses were performed using a Waters/Micromass (Manchester, UK) ZQ mass spectrometer coupled to a Waters (Milford, MA USA) model 2690 HPLC pump. A Superspher 100 RP-18 column (250 × 2 mm) was used.

### Chemicals

All cell culture material and other chemicals, if not indicated otherwise, were purchased from Sigma-Aldrich (St. Louis, MO, USA). Ramentaceone was dissolved in DMSO for the treatment of cells (final concentration in medium was 0.5%).

### Cell Culture

The BT474, SKBR3, MCF-7 and MDA-MB-231 breast cancer cell lines were purchased from Cell Line Services (Germany). SKBR3, MCF-7 and MDA-MB-231 cells were cultured in DMEM medium, BT474 cells were cultured in DMEM/F12 medium. Media were supplemented with 10% fetal bovine serum, 2mM glutamine, 100 units/mL penicillin and 100 μg/mL streptomycin. Cultures were maintained in a humidified atmosphere with 5% CO_2_ at 37°C in an incubator (Heraceus, Hera cell).

### Cytotoxicity Assay

The viability of cells was determined using the MTT [(3-(4,5-dimethylthiazol-2-yl)-2,5-diphenyltetrazolium bromide] assay. Cells were treated with ramentaceone (0–15 μM) for 24 h. Analysis was performed according to the previously published procedure [12].

### Clonogenicity Assay

To determine long-term effects of ramentaceone on BT474 and SKBR3 cells, cells were seeded in 6-well plates (10^3^ cells/well) and treated with ramentaceone (0–15 μM) for 3 h. The medium was discarded and fresh medium was added to the wells, after which cells were allowed to grow for 16 days to form colonies and stained with crystal violet (0.5%).

### Caspase Activity Determination

To examine the induction of caspase activity by ramentaceone, the FLICA Apoptosis Detection Kit (Immunochemistry Technologies) was used. The kit uses FLICA (Fluorochrome Inhibitor of Caspases), a carboxyfluorescein-labeled fluoromethyl ketone peptide, which irreversibly binds to many active caspases. Caspase labeling was performed according to the manufacturer’s instructions. Briefly, cells were treated with ramentaceone (0–15 μM) for 12 h after which they were collected and suspended in a buffer containing the caspase inhibitor. After a 1 h incubation at 37°C under 5% CO_2_ cells were washed with washing buffer and the fluorescence intensity of fluorescein was determined with flow cytometry (BD FACSCalibur). Caspase activity was determined as the amount of fluorescence emitted from FLICA probes bound to the caspases.

### Annexin V-PE staining

Apoptosis induction was detected with an Annexin V-PE Apoptosis Detection Kit I (BD Biosciences, Belgium) according to the manufacturer’s instructions. Briefly, cells were treated with ramentaceone (0–15 μM) for 24 h, after which cells were collected, washed with Annexin-binding buffer, and stained with Annexin V- phycoerythrin (PE) and 7-amino-actinomycin (7-AAD). After incubation at 15°C for 15 min in the dark, samples were analyzed by flow cytometry (BD FACSCalibur)

### Western Blot Analysis

Western blot analysis was performed according to the previously published procedure [12]. Cells were treated with ramentaceone (0–15 μM) for 24 h or were pre-treated with the PI3K inhibitor, LY294002 (5 μM) and subsequently treated with 5 μM ramentaceone for 24 h. Specific primary antibodies: anti-β-actin (1:1000) (Cell Signaling, Germany), anti-Bax, anti-Bak, anti-Bcl-2 (1:250) (Santa Cruz, Heidelberg, Germany), anti-cleaved caspase-3 (Asp175) (1:1000) (Cell Signaling, Germany), anti-cleaved PARP (Asp214), anti-PI3K p85, anti-phospho-PI3K p85 (Tyr458)/p55 (Tyr199), anti-Akt, anti-phospho-Akt (Ser473) (1:1000) (Cell Signaling, Germany) were incubated with membranes overnight at 4°C. Membranes were further incubated at room temperature for 1 h with HRP-conjugated secondary antibodies (Cell Signaling, Germany) and proteins were detected by chemiluminescence (ChemiDoc, Bio-Rad) with a HRP substrate (Pierce).

### PI3-kinase activity assay

In order to detect and quantify PI3-kinase activity the Amplified Luminescent proximity Homogenous Assay (AlphaScreen) technology was employed using the PI3-kinase kit (K-1300), Echelon, USA). The binding reaction of a biotynylated-PI(3,4,5)P_3_ probe to a PIP(3,4,5)P_3_ detector GST-fusion protein was detected using the AlphaScreen GST detection kit (PerkinElmer) comprising Donor beads conjugated with streptavidin and Acceptor beads conjugated with anti-GST. During the assay, interactions between biotynylated-PI(3,4,5)P_3_ and PI(3,4,5)P_3_ binding protein bring the Acceptor and Donor into close proximity and upon the excitation of the Donor beads an amplified AlphaScreen signal is generated. Enzymatic reactions were performed according to manufacturer’s instructions in 384-well white optiplates (PerkinElmer, Germany) in a final volume of 25 μl per well. Reaction mixtures contained ramentaceone (100 μM—0.01 nM) or LY294002 (100 μM—0.01 nM), 10 μM ATP, 5 μM PIP_2_ substrate and 25 ng PI3-kinase (E-2000, Echelon Biosciences) in a reaction buffer (2.5 mM MgCl_2_, 5 mM HEPES, pH 7.4). Reactions were carried out for 1 h at room temperature after which 10 nM biotinylated-PIP_3_, in a detection buffer (10 mM Tris, pH 7.4, 150 mM NaCl, 1 mM DTT, and 0.1% Tween-20), was added. This was followed by the addition of l0 nM PIP_3_ binding protein and 20 μg/ml of both AlphaScreen Donor and Acceptor beads (AlphaScreen GST Detection Kit, PerkinElmer, Germany). Plates were incubated for 2 h after which luminescence was measured with an EnVision Multilabel plate reader (PerkinElmer Germany).

### Akt knockdown

The expression of Akt was silenced in BT474 and SKBR3 cells using Akt1, Akt2 and Akt3 siRNA and control, scrambled siRNA (Santa Cruz, Germany). Cells were transiently transfected with Akt or control siRNA according to the manufacturer’s instructions and 24 h post-transfection, cells were either collected for Western blot analysis or treated with ramentaceone.

### Statistical analysis

Values are expressed as mean ± SD of at least three independent experiments. Statistical analysis was performed using GraphPad Prism 5.0 (GraphPad software). Differences between control and ramentaceone-treated samples were analyzed by one-way ANOVA with Tukey's post-hoc tests. Differences between single agent and double agent treatments were analyzed by two-way ANOVA with Bonferroni post-tests. A *p* value of <0.05 was considered as statistically significant in each experiment. Statistical analysis of IC_50_ values were calculated from concentration-response curves using GraphPad Prism 5.0 (GraphPad Software) with the equation: Y = Bottom + (Top-bottom)/1 + 10LogEC50-X.

## Results

### Antiproliferative effects of ramentaceone towards breast cancer cells

The effects of ramentaceone (Fig 1) on the proliferation of breast cancer cells were determined with the use of the MTT assay. HER2-positive (BT474 and SKBR3) and HER2-negative (MCF-7 and MDA-MB-231) breast cancer cells were treated with increasing concentrations of ramentaceone. Ramentaceone inhibited the proliferation of the examined cell lines in a dose-dependent manner (Fig 2A), however, higher activity was observed towards the HER2-overexpressing cell lines, BT474 and SKBR3. After a 24 h treatment with ramentaceone, the obtained IC_50_ values for HER2-positive, BT474 and SKBR3, cells were 4.5 ± 0.2 μM and 5.5 ± 0.2 μM, respectively, whereas for the HER2-negative, MDA-MB-231 and MCF-7, cells IC_50_ values of 7 ± 0.3 μM and 9 ± 0.4 μM were obtained. Since ramentaceone exhibited higher activity towards HER2-positive cells, long-term effects of ramentaceone on proliferation and colony formation of these cells were determined with the use of the colony forming assay. Ramentaceone inhibited colony formation of BT474 and SKBR3 cells in a concentration-dependent manner. At the concentration of 0.5 μM, ramentaceone inhibited colony formation of BT474 and SKBR3 cells by 70 and 60%, respectively, whereas at 2.5 μM colony formation was inhibited by 100% in both cell lines (Fig 2B). Results of the clonogenic assay have been shown to correlate well with tumorgenicity analysis in vivo [13]. Moreover, analysis performed using samples from breast cancer patients showed that the clonogenic assay predicted the clinical response toward several agents [14], indicating the potential of ramentaceone in HER2-positive breast cancer therapy.

**Fig 1:** Structure of ramentaceone (5-hydroxy-7-methyl-1,4-naphthoquinone).

**Fig 2:** Effects of ramentaceone on the viability of breast cancer cells. (A) Cytotoxic activity of ramentaceone toward HER2-overexpressing (BT474 and SKBR3) and HER2-negative (MCF-7 and MDA-MB-231) breast cancer cells. Cells were treated with ramentaceone (0–15 μM) for 24 h and cell survival was assessed with the MTT assay (n = 3). (B) Influence of ramentaceone on clonogenicity of HER2-positive breast cancer cells, SKBR3 and BT474. Cells were treated with ramentaceone (0–15 μM) for 3 h and allowed to grow for 16 days to form colonies. Values represent mean ± SD of three independent experiments. *p* < 0.05 (*) indicates differences between control and ramentaceone-treated cells.

### Inhibition of the PI3K/Akt signaling pathway by ramentaceone in breast cancer cells

To elucidate the mechanism of ramentaceone-induced cell death, the involvement of ramentaceone in PI3K/Akt signaling was examined. Breast cancer cells were treated with ramentaceone in the concentration range of 0–15 μM for 24 h and the levels of proteins involved in PI3K/Akt signaling were examined. Western blot analysis showed that treatment with ramentaceone reduced the expression of the regulatory subunit of the PI3K (p85) protein in cells in a dose dependent manner. Further analysis was carried out to determine the influence of ramentaceone on the phosphorylation of the Akt protein. Western blot analysis revealed inhibition of Akt phosphorylation upon ramentaceone treatment as shown by a decrease in the levels of phosphorylated Akt at Ser 473. The levels of phosphorylated Akt decreased in a concentration-dependent manner upon ramentaceone treatment with no change in the expression of total Akt (Fig 3A). Due to the higher inhibitory activity of ramentaceone towards HER2-positive cells, a time course analysis of PI3K and p-Akt inhibition by ramentaceone was further examined in these cells. Cells were treated with 5 μM of ramentaceone for 1, 6 and 12 h, after which PI3K and p-Akt levels were determined with Western blot analysis. A significant decrease in PI3K and p-Akt levels were observed 1 h post-ramentaceone treatment and decreased in a time-dependent manner in SKBR3 and BT474 cells (Fig 3B). To further evaluate the ability of ramentaceone to inhibit PI3K activity, a kinase assay employing AlphaScreen technology was used. Ramentaceone was examined in the concentration range of 100 μM—0.01 nM for 1 h. The PI3K inhibitory activity of ramentaceone was compared to that of the PI3K inhibitor, LY294002, which was examined in the same concentration range. As shown in Fig 4, ramentaceone inhibited PI3-kinase activity with an IC_50_ value of 2 ± 0.3 μM, higher than that of LY294002 (IC_50_ 4 ± 0.3).

**Fig 3:** Effects of ramentaceone on the expression levels of PI3K/Akt signaling proteins. (A) Concentration-dependent inhibition of PI3K/Akt signaling. Breast cancer cells were treated with ramentaceone (0–15 μM) for 24 h and the levels of PI3K p85, phospho-PI3K p85 (Tyr458)/p55 (Tyr199), phospho-Akt (Ser 473), and Akt were assessed by Western blot analysis. (B) Time-dependent inhibition of PI3K/Akt signaling. BT474 and SKBR3 cells were treated with ramentaceone (5 μM) for the indicated time periods and the levels of PI3K p85, phospho-Akt (Ser 473), and Akt were assessed by Western blot analysis. Protein levels were determined by densitometric analysis. Values represent mean ± SD of three independent experiments. *p* < 0.05 (*) indicates differences between control and ramentaceone-treated cells.

**Fig 4:** Inhibition of phosphoinositide-3-kinase (PI3-kinase) activity by ramentaceone in breast cancer cells. The AlphaScreen technology was used to determine enzyme activity. The AlphaScreen assay was performed with ramentaceone or LY294002, added at concentrations ranging from 100 μM to 0.01 nM, 25 ng PI3-kinase, 5 μM PIP_2_, 10 μM ATP and with an incubation time of 1 h. Values represent mean ± SD of three independent experiments.

### Induction of apoptosis by ramentaceone in breast cancer cells

The ability to induce apoptosis in cancer cells is a desired feature of a potential chemotherapeutic agent. To determine whether ramentaceone induces apoptotic-mediated cell death in breast cancer cells a characteristic feature of apoptotic cell death, namely phosphatidylserine externalization, was analyzed in ramentaceone-treated cells. Cytometric analysis of cells stained with Annexin V-PE revealed a dose-dependent increase in apoptosis induction in HER2-positive and HER2-negative breast cancer cells. In accordance to the results of the MTT assay, the HER2-positive cells were more sensitive to ramentaceone-induced cell death. At the concentration of 5 μM the percentage of BT474 apoptotic cells increased 3-fold and at 15 μM, 6-fold, whereas in SKBR3 cells the percentage of apoptotic cells increased 1.5-fold at 5 μM and at 15 μM, 3-fold (Fig 5).

**Fig 5:** Induction of apoptosis by ramentaceone in breast cancer cells. Apoptotic changes in plasma membrane induced by ramentaceone. Cells were treated with ramentaceone (0–15 μM) for 24 h, stained with Annexin V-PE/7-AAD, and analyzed by flow cytometry. Values represent mean ± SD of three independent experiments. *p* < 0.05 (*) indicates differences between control and ramentaceone-treated cells.

The influence of ramentaceone on downstream targets of the Akt protein, the Bcl-2 family proteins, was further examined. The levels of pro-apoptotic Bax and Bak proteins and anti-apoptotic Bcl-2 protein were examined in ramentaceoone-treated HER2-positive breast cancer cells. BT474 and SKBR3 cells were treated for 24 h with ramentaceone and Western blot analysis was performed in order to verify protein levels of Bax, Bak and Bcl-2. Our research showed that ramentaceone increased the levels of pro-apoptotic Bax and Bak proteins in a concentration-dependent manner. Furthermore, ramentaceone decreased the levels of anti-apoptotic Bcl-2 in both SKBR3 and BT474 cells in a dose-dependent manner (Fig 6A). The effects of ramentaceone on caspase activation were subsequently examined. BT474 and SKBR3 cells were treated for 12 h with ramentaceone, after which cytometric analysis was performed. The results revealed a dose-dependent increase in ramentaceone-induced caspase activation. At the concentration of 5 μM the percentage of apoptotic BT474 cells increased 3-fold in comparison with the control and at 15 μM caspase activation increased 5-fold. In SKBR3 cells the percentage of apoptotic cells increased 2-fold and 4-fold at the concentrations of 5 μM and 15 μM, respectively (Fig 6B). The results of caspase activation were confirmed by showing a ramentaceone-induced, dose-dependent increase in caspase-3 activation and PARP cleavage with Western blot analysis (Fig 6C).

**Fig 6:** Effects of ramentaceone on expression levels Bcl-2 family proteins and caspase activity in breast cancer cells. (A) Effects of ramentaceone on the expression levels of Bax, Bak and Bcl-2 in SKBR3 and BT474 cells. Cells were treated with ramentaceone (0–15 μM) for 24 h, and the levels of Bax, Bak, Bcl-2 were assessed by Western blot analysis. Protein levels were determined by densitometric analysis (B) Induction of caspase activity in BT474 and SKBR3 cells. Cells were treated with ramentaceone (0–15 μM) for 12 h, and enzyme activity was determined by flow cytometry with the use of a caspase inhibitor, FAM-VAD-FMK (C) Activation of caspase-3 and cleavage of PARP by ramentaceone in BT474 and SKBR3 cells. Cells were treated with ramentaceone (0–15 μM) for 24 h, and the levels of cleaved caspase-3 and PARP were assessed by Western blot analysis. Protein levels were determined by densitometric analysis. Values represent mean ± SD of three independent experiments. *p* < 0.05 (*) indicates differences between control and ramentaceone-treated cells.

### Role of PI3K/Akt inhibition in ramentaceone-mediated apoptosis induction

Since ramentaceone was shown to inhibit PI3K/Akt signaling, the role of PI3K and Akt inhibition in ramentaceone-induced apoptosis was examined. A PI3K inhibitor, LY294002, was used to determine the role of PI3K in ramentaceone-mediated apoptosis induction. For this purpose HER2-overexpressing cells were pre-treated with LY294002 for 1 h after which cells were exposed to 5 μM of ramentaceone for 24 h. Western blot analysis showed that pre-treatment of cells with the PI3K inhibitor decreased the levels p-Akt in BT474 and SKBR3. Moreover, the combination of LY294002 and ramentaceone significantly induced the levels of downstream Akt targets, Bax and Bak and downregulated anti-apoptotic Bcl-2 in comparison with single-agent treated cells (Fig 7). To further verify the involvement of Akt in ramentaceone-induced apoptosis, Akt expression was transiently silenced in HER2-overexpressing breast cancer cells. BT474 and SKBR3 cells were transiently transfected with Akt siRNA or control, scrambled siRNA and 24 h after transfection Western blot analysis was performed in order to determine Akt levels in cells. As shown in Fig 8A, Akt expression was reduced with Akt siRNA in BT474 and SKBR3 cells in comparison with cells transfected with the control, scrambled siRNA. To determine the influence of Akt on ramentaceone-mediated apoptosis induction, 24 h after transfection BT474 and SKBR3 cells were treated with ramentaceone (5 μM) for 24 h and Annexin V-PE straining was performed. The silencing of Akt in BT474 and SKBR3 cells increased the percentage of the apoptotic cell population (early and late apoptotic) in comparison with the control population, transfected with control siRNA. Furthermore, treatment with ramentaceone significantly increased apoptosis induction in cells with Akt knockdown in comparison with control cells. Akt silencing increased ramentaceone-induced apoptosis in BT474 and SKBR3 cells by 25% and 15% (Fig 8B), respectively. The results obtained with PI3K inhibition and Akt silencing indicate the involvement of PI3K/Akt signaling in ramentaceone-mediated apoptosis induction.

**Fig 7:** The role of PI3K inhibition in ramentaceone-mediated apoptosis induction. BT474 and SKBR3 cells were pre-treated with the PI3K inhibitor LY294002 (5 μM) after which cells were treated with ramentaceone (5 μM) for 24 h. Bax, Bak, Bcl-2 levels were assessed by Western blot analysis. Protein levels were determined by densitometric analysis. Values represent mean ± SD of three independent experiments. *p* < 0.05 (*) indicates differences between control and ramentaceone-treated cells. *p* < 0.05 (#) indicates differences between ramentaceone-treated and LY294002 pre-treated samples.

**Fig 8:** The role of Akt inhibition in ramentaceone-mediated apoptosis induction. (A) Silencing of Akt by siRNA in BT474 and SKBR3 cells. Cells were transiently transfected with Akt siRNA and 24 after transfection, Akt silencing was confirmed with Western blot analysis. (B) Induction of apoptosis by ramentaceone in cells transfected with Akt siRNA and control siRNA. 24 h after transfection cells were treated with ramentaceone (5 μM) for 24 h, stained with Annexin V-PE/7-AAD, and analyzed by flow cytometry. Representative of three independent experiments. *p* < 0.05 (*) indicate differences between control siRNA and Akt siRNA transfected cells treated with ramentaceone.

## Discussion

The phosphoinositide 3-kinase (PI3K) signaling pathway is of central importance in breast cancer and plays an important role in processes critical for cancer progression including proliferation, survival, motility, angiogenesis and metabolism. Hyperactivation of PI3K/Akt signaling has been associated with an altered response of cancer cells to therapy such as chemotherapy and radiation [15]. PI3K/Akt signaling lies downstream of receptor tyrosine kinases and is activated by the binding of various growth factors to their cognate receptors. Growth factor binding activates the lipid kinase PI3K, a heterodimer comprising a regulatory p85 and catalytic p110 subunit, which catalyzes phosphatidylinositol-3,4,5-triphosphate (PIP3). This triggers the attachment of Akt to the plasma membrane resulting in Akt activation through phosphorylation at two sites, Thr308 and Ser473 [16]. Akt plays a central role in apoptosis inhibition through its regulatory effects on various downstream targets such as the Bcl-2 family proteins. Akt directly phosphorylates the protein Bad of the Bcl-2 protein family. Bad is a pro-apoptotic protein, which associates with anti-apoptotic Bcl-2 and blocks Bcl-2 from binding with pro-apoptotic Bcl-2 family members such as Bax and Bak. The phosphorylation of Bad by Akt allows the binding of Bad to 14-3-3 proteins, therefore enabling anti-apoptotic Bcl-2 to bind to pro-apoptotic Bcl-2 family members, Bax and Bak, suppressing Bad-induced apoptosis [17]. In accordance with these findings, our research revealed that ramentaceone inhibits PI3K/Akt signaling though downregulating PI3K kinase and inhibiting Akt phosphorylation. Furthermore, ramentaceone induces apoptosis through targeting downstream effectors of the Akt protein, namely proteins of the Bcl-2 family. An increase in the levels of pro-apoptotic proteins Bax and Bak were observed, concomitant with a decrease in anti-apoptotic Bcl-2. The role of PI3K/Akt inhibition in ramentaceone-mediated apoptosis induction was shown by an increase in apoptosis induced by ramentaceone in cells pretreated with a PI3K inhibitor, LY294002. This was further confirmed by silencing the expression of Akt in breast cancer cells with Akt siRNA and showing that knockdown of Akt increases the sensitivity of BT474 and SKBR3 cells towards ramentaceone. These results confirm that ramentaceone induces apoptosis through PI3K/Akt inhibition in breast cancer cells.

PI3K/Akt activation renders breast cancer cells resistant to apoptosis, which is a major barrier in efficient breast cancer treatment [18]. In particular PI3K/Akt upregulation confers resistance of HER2-overexpressing breast cancer cells to apoptosis induced by HER2- directed therapy. In many studies apoptosis was found to be enhanced in HER2-positive cells through targeting down-stream effectors of the PI3K/AKT signaling pathway. In addition, the inhibition of PI3K/Akt signaling components has been shown to enhance HER2-targeted therapy. PI3K inhibition along with HER2-targeted drugs has been shown to reduce tumor cell growth more significantly than either drug alone [19]. Similarly, Bcl-2 inhibitors have been found to increase lapatinib efficiency in HER2-positive cells [20]. Furthermore, targeting PI3K signaling components has been found to reverse resistance acquired toward HER2-directed therapy. Increased Bcl-2 expression has been associated with resistance to trastuzumab. The study of Crawford and Nahta et al [4]. showed that trasuzumab resistant cells displayed higher sensitivity to the Bcl-2 inhibitor, ABT-737, than parental cells. Moreover, the combination of ABT-737 and trastuzumab was found to inhibit the growth of trastuzumab-resistant cells more significantly than either drug alone [4]. Similarly, the Akt inhibitor, triciribine, in combination with trastuzumab caused a synergistic reduction of traztuzumab-resistant tumor growth [21]. The application of trastuzumab along with a PI3K inhibitor, SF1126, also induced a synergistic effect toward trastuzumab-resistant cells [22]. These findings point to the importance of targeting multiple components of the PI3K/Akt pathway as means of improving therapy response and combating drug resistance. Our research revealed that ramentaceone downregulates components of the PI3K/Akt pathway associated with HER2-targeted drug resistance. This points to the promising potential of ramentaceone in HER2-positive breast cancer therapy in particular adjuvant therapy.

Compounds comprising a quinone moiety are one of the largest groups of compounds used in anticancer therapy [23]. Naphthoquinones in particular have gained interest as potential anticancer agents [24–27]. Plumbagin, an extensively researched naphthoquinone, has been shown to exert significant anti-proliferative and anti-cancer activity in various animal models and cancer cell lines [28–30], including breast cancer [31–33]. Studies performed by Kuo et al. [34] showed that plumbagin significantly reduced the size of MDA-MB-231 tumor xenografts by 70% in mice without toxic side-effects. Our previous research revealed high antiproliferative activity of plumbagin towards HER2-overexpressing breast cancer cells [27]. The results presented herein show that ramentaceone exerts higher anti-clonogenic and pro-apoptotic activity towards HER2-overexpressing breast cancer cells in comparison with plumbagin. Due to the structural similarity of these compounds, further research into the activity of ramentaceone toward breast cancer is warranted.

In conclusion, our research shows that ramentaceone induces apoptosis through inhibiting PI3K/Akt signaling. Ramentaceone reduced PI3K expression, suppressed Akt phosphorylation and inhibited downstream targets of Akt, such as the anti-apoptotic protein Bcl-2 and increased the expression of pro-apoptotic Bax and Bak. Our findings provide a rationale for further research on ramentaceone as a potential agent in the treatment of breast cancer, in particular HER2-overexpressing breast cancer.
